RETRACTED

# A novel study on the influence of graphene-based nanofluid concentrations on the response characteristics and surface-integrity of Hastelloy C-276 during minimum quantity lubrication

**DOI:** 10.1016/j.heliyon.2023.e19175

**Published:** 2023-08-22

**Authors:** Gurpreet Singh, Shubham Sharma, A.H. Seikh, Changhe Li, Yanbin Zhang, S. Rajkumar, Abhinav Kumar, Rajesh Singh, Sayed M. Eldin

**Affiliations:** a Department of Mechanical Engineering, I.K. Gujral Punjab Technical University, Kapurthala, Punjab, India; b Department of Mechanical Engineering, Chandigarh University, Gharuan, Mohali, Punjab, India; c Mechanical Engineering Department, University Center for Research & Development, Chandigarh University, Mohali, Punjab, 140413, India; d School of Mechanical and Automotive Engineering, Qingdao University of Technology, 266520, Qingdao, China; e Mechanical Engineering Department, College of Engineering, King Saud University, P.O. Box 800, Riyadh, 11421, Saudi Arabia; f Department of Mechanical Engineering, Faculty of Manufacturing, Institute of Technology, Hawassa University, Ethiopia; g Department of Nuclear and Renewable Energy, Ural Federal University Named After the First President of Russia, Boris Yeltsin, 19 Mira Street, 620002, Ekaterinburg, Russia; h Uttaranchal Institute of Technology, Uttaranchal University, Dehradun, 248007, India; i Department of Project Management, Universidad Internacional Iberoamericana, Campeche, C.P., 24560, Mexico; j Center of Research, Faculty of Engineering, Future University in Egypt, New Cairo, 11835, Egypt

**Keywords:** Hastelloy C-276, Graphene nanoparticle, Scanning electron microscopy, Surface roughness, Concentration

## Abstract

In present investigation, the impact of nanoparticle concentration on the machining accomplishment of Hastelloy C-276 has been examined in turning operation. The outputs like temperature, surface roughness, chip reduction coefficient (CRC), tool wear, and friction coefficient along with angle of shear have been estimated. The graphene nanoparticles (GnP) have been blended into soybean oil in distinct weight/volume ratio of 0.5, 1 and 1.5%. The experimental observations revealed that higher concentration of nanoparticles has enhanced the heat carrying capacity of amalgamation by 12.28%, surface roughness (27.88%), Temperature (16.8%), tool wear (22.5%), CRC (17.5%), coefficient of friction (46.36%) and shear angle (15%). Scanning electron microscopy identified nose wear, abrasion, adhesion and loss of tool coating. Further, lower tool wear has been noticed at 1.5% concentration, while the complete failure of insert has been reported during 116 m/min, 0.246 mm/rev having 0.5% concentration. ANOVA results exhibited that surface roughness is highly influenced by speed rate (41.66%) trailed by feed rate (28.16%) and then after concentration (13.68%). Temperature is dominated by cutting speed (69.31%), concentration (14.53%) and feed rate (13.25%). Likewise, tool wear was majorly altered by cutting speed (67.2%) accompanied by feed rate (23.90%) and thirdly concentration of GnP (5.03%).

RETRACTED

## 1 Introduction

In this era of industrialization machining of Ni based alloy is gaining popularity by virtue of having magnificent mechanical and thermal properties. This makes superalloys suitable for various applications like aerospace, chemical plants, nuclear reactor components and petroleum industry equipment. The conventional flood lubrication of superalloy is not viable due to environmental issues, cost of wastage disposal, health hazards and costly recycling set up. On the other side, the dry machining of such material is not feasible at higher cutting speed because of quick tool failure and lower surface characteristics. Further, the cryogenic cooling of various super alloys has been practiced these days to extend the tool life along with excellent surface quality but limited due to higher cost of cryogenic liquid and sometimes cold cracking of machine surface. Therefore, minimum quantity lubrication (MQL) should be the possible solution for the machining of superalloy. Also, the addition of nano-fluids to MQL lubricant reduces the heat formation, surface irregularities and tool life should be enhanced that provide economic machining than conventional flood cooling and dry machining. The examination on the addition of aluminum oxide nano-particles to MQL fluids while turning of Ni–Cr alloy (718) has reduced the insert damage and friction coefficient because of wetting properties [1]. The exploration on the performance of AISI 1045 utilizing MQL revealed that forces and temperature were minimized with variation in MQL cone angles [2]. The investigations on the machining of Hastelloy-X in dry and nano MQL was conducted and revealed that 0.25% concentration of hBN fluid has improved the performance [3]. The superalloys having constitutes of Ni are suitable for high temperature application because of higher thermal stability and prevention against corrosion [4]. These superalloys are mainly (50%) utilized in aerospace, furnace components, superconductivity elements and chemical industries due to their FFC structure. The addition of Cr and Mo with more than 30% of weight extends their wear, oxidation and low cracking tendency. Consequently, amalgamation of W, Co and Fe in single solution element leads to higher mechanical strength along with extensive temperature stability [[5], [6], [7], [8]]. The investigations on crack propagations, corrosion, cyclic fatigue and hot machinability characteristics of Hastelloy-X have been initiated [[9], [10], [11]]. The utility of bio based oil MQL have greater machining output compared to conventional cutting fluids, however it has limited thermal stability than former [12]. The problem of thermal instability can be refined with addition of nanofluids (MOS_2_) to bio-oil and thus enhance the tribo characteristics too [13,14]. MQL machining performance of Ni based alloy using amalgamation of aluminium oxide nano-fluids truncated the forces, heat formation, roughness and flank damage [15]. The lower lubricant usage (6-times) than traditional system is the significant feature of MQL machining [16]. The utility of PVD coating under electrostatic extreme velocity MOS_2_ lubricant has lowered tool wear than flood and dry system [17]. The modified Jathpora oil MQL turning of Mg–Si based alloy revealed the significant improvement in force and surface roughness in contrast to mineral oil [18]. Implementation of crystalline non cellulose nanofluids has improved the thermal conductivity, viscosity and further reduced the temperature at tool chip point [19]. The research on the machining forces, temperature and residual stresses of Ni based 718 alloy using TiO_2_ nano-lubricant reported minimization of listed outcomes compared to conventional system [20]. Review on the capability of nano-cutting fluids MQL machining listed the multiple advantages compared to traditional ways assuming surface quality, wear, heat generation and friction coefficient [21]. The impact of mixing carbon nano tube to SAE20W40 oil during machining of stainless steel reported enhancement of tool wear due to better penetration and significant lubrication action [22]. The comparison on the machining output of grinding Inconel 718 using graphene based MQL with dry and oil based machining pointed out that MQL machining exhibited superior outcomes considering surface finish, heat generation and operating forces [23]. While turning the material with silver based nanofluids the performance parameter like forces, temperature and roughness were reduced [24]. Likewise, temperature, forces and surface irregularities were enhanced for Ti alloy cutting using MQL [25]. The utility of GnP-MQL in orthogonal machining of carbon steel mentioned the decrease in forces, surface waviness and tool erosion than flood condition [26]. The study on the mechanics of machining and specimen quality while roughing the Ni–Cr steel using MQL has been conducted [27]. The comparison of alumina and MoS_2_ nano-fluids with Al_2_O_3_ was performed and revealed that rise in concentration of nano-fluids during machining of AISI 304 minimized the temperature and tool damage [28]. The analysis of machining Mg alloys assisted with MQL revealed the minimization of machining force, tool erosion, surface waviness and temperature w.r.t dry condition [29]. The use of Al_2_O_3_ nano lubricant as cutting oil has provided the magnificent performance during turning of Ti alloys by reducing the power consumption, wear rate of tool and roughness of machined component [30]. The multi-walled carbon nanotubes employed for turning of Ni–Cr alloys minimized the tool wear because of excellent cooling ability as compared to aluminum oxide nano fluids [31]. In an another study on machining of Ti alloy confirmed that vegetable oil MQL mixed with 2% of carbon nano-fluids minimized the specific power consumption and tool wear appreciably compared to Al_2_O_3._ In addition to this, blending of 4% CNT to lubricant has lowered the texture of specimen during turning of Ti alloys [32]. Usage of graphene and silicon dioxide dual nano-fluids for milling of austenitic steel revealed the shrinkage of friction coefficient because of covering layer formation [33]. The capability of AISI 1045 implementing minimal lubricant quantity with graphite explored the reduction of heat and surface waviness [34]. The surface quality of work item was enhanced during grinding of Nickel based alloys cooled with Al_2_O_3_ and silicon dioxide nanoparticle [35]. The output of turning AISI 304 with alumina-graphene nano lubricants explored the miniature of surface irregularities, forces and feed forces [36]. The minimization of surface quality during nano MQL of Cu w.r.t dry and oil lubrication of H11 steel turning has been reported [37]. Utilization of Al_2_O_3_ nano fluid MQL for turning of Inconel 600 alloy observed the decrement in roughness, tool damage and heat generation compared to vegetable oil MQL [38]. The outcomes of AISI 1060 machining in dry and lubricant with least proportion situation find out the better responses in MQL [39]. The investigation on output of turning EN-31 Steel with traditional cutting fluids, mineral oil and CNT revealed the better performance in case of CNT compared to other conditions [40]. The MQL machining of TiO_2_ nano-fluids reported the decrease in heat formation during milling of AA6061 because of larger heat extraction, low adhesion and edge reliability of TiO_2_ [41]. The comparison of heat absorption capacity in different nano-fluids like SiO_2_, Al_2_O_3_ and TiO_2_ blended with vegetable oil revealed that gain in agglomeration of nanoparticles enhance the heat carrying capacity. Further, SiO_2_ was found with highest specific heat compared w.r.t other nano-fluids [42]. Machining capability of distinct nano-fluids in grinding of alloy (Ni) reported that CNT based MQL has reduced the surface roughness due to minor contact angle and surface tension [43]. MQL is becoming promising solution to dry and conventional lubrication ways due to lower friction coefficient by discharging minute amount of cutting fluid at smaller contact zone of machining [44]. The various researches suggested that using MQL can enhance the cutting point life, surface texture, temperature and cutting stresses while machining different grades of steel and super alloys [[45], [46], [47], [48], [49], [50]]. On the other hand, in certain cases, the performance of MQL has been found limited cooling ability during processing of difficult to cut materials. Therefore, addition of other media is required to achieve excellent cooling action along with good lubricity of MQL. Hence mixing of nanoparticle of different nature with least lubricant amount has gained momentum in current paradigm of industry 4.0. It has extended the tool life as well surface quality [51]. The thermal analysis of palm oil MQL blended with 6 types of nano-fluids such as greasy, ceramics, carbon as well composite types observed that addition of nano-fluids enhanced the heat conduction and viscous effect of base fluid. Consequently, the cutting forces and temperature was turn down. Further, highest heat carrying capacity was noticed in CNT [52]. The significance of nano particle agglomeration in MQL assisted minute drilling revealed that power consumption and torques were lowered [53]. Machining forces and finish of work in hard turning of 90CrSi utilizing different nano fluids mixed with soybean and water emulsion concluded that nanofluids and its concentration have influenced the performance [51].

RETRACTED

### 1.1 Research objectives

The review of literature indicates that the investigation on the machining of Hastelloy C-276 has been rarely reported using different concentration of nanoparticles mixed with lubrication oil. Further, the tool wear during machining of this material using graphene nano fluids with different concentration has been investigated rarely. The main aim of present research is to examine the impact of concentration on various output responses. Therefore, the current investigations will provide suitable data for future studies and industries involved with manufacturing of super alloys products.

## 2 Material and methods

Experiments have been carried out on Ni based superalloy C-276 rods of 0.052 m diameter and 0.550 m long. The details of input variables like speed, feed and cooling conditions have been explored in Table 1 keeping constant doc 0.5 mm for all trials. The MQL mist of graphene-soybean oil mixtures of different concentration have been applied through single nozzle focused on rake part of tool at margin of 30 mm having angle of 45°. The flow of MQL mixture has been fixed to 20 ml/h at pressure of 4 bar. The properties of pure Soybean oil and mixture of different concentration have been listed in Table 2. The workpiece has higher heat carrying capacity making it suitable for heat resistant applications, but lower thermal conductivity creates the machining difficult that impact the tool life and surface quality. It contains 57.9% of nickel, 16% molybdenum, 15.4% of chromium, 5.5% of iron, and 3.7% of tungsten. In addition, minor content (less than 1%) of silicon, carbon, phosphorus, cobalt enhance the properties of this super alloys. As far as physical, mechanical and thermal properties are concerned, it has density of 889 kg/m^3^, hardness 87 HRB, Elastic modulus 205 GPa, Sp. Heat 427 J/kg°C and conductivity (thermal) 10.5 W/m°C. For experimentation, three levels, three factors of input variables along with four output parameters have been listed in Table 3 leading to total 27 experiments.

**Table 1:** Factor information.

Factor	Units	Minimum Level (−1)	Medium Level (0)	High Level (1)	Output Responses
Cutting Speed (A)	m/min	51	82	116	Surface roughness (Ra), Cutting temperature (°C), Tool wear (mm), CRC
Feed rate (B)	mm/rev	0.06	0.112	0.246	
Nanoparticle concentration (C)	Wt/v. %	0.5	1	1.5

**Table 2:** Important properties of Lubricant and mixtures.

Properties	Pure Soybean oil	0.5% GnP	1% GnP	1.5% GnP
Flash point	240 °C	248 °C	252 °C	258 °C
Specific gravity	0.910	0.916	0.926	0.932
Kinematic viscosity @ 40 °C (cSt)	33.2	33.7	34.2	34.8
Thermal conductivity (W/mk)	0.171	0.178	0.183	0.192

**Table 3:** Details of input variables and experimental results.

S.N	Input variables			Output responses			
	Cutting speed (m/min)	Feed rate (mm/rev)	N.C wt./vol. (%)	S.R (Ra, μm)	Cutting temperature (°)	Tool wear (mm)	CRC
1	51	0.06	0.5	0.68	146	**0.186**	2.20
**2**	**51**	**0.06**	**1**	**0.65**	**138**	**0.172**	**2.17**
3	51	0.06	1.5	0.69	126	0.144	2.14
4	51	0.112	0.5	0.72	158	0.226	2.06
5	51	0.112	1	0.68	150	0.218	1.72
6	51	0.112	1.5	0.74	132	0.204	1.69
7	51	0.246	0.5	0.78	163	0.258	1.95
8	51	0.246	1	0.71	158	0.232	1.83
9	51	0.246	1.5	0.68	140	0.224	1.75
10	82	0.06	0.5	0.61	162	0.196	2.67
11	82	0.06	1	0.58	157	0.188	2.64
12	82	0.06	1.5	0.54	149	0.184	2.57
13	82	0.112	0.5	0.65	172	0.266	1.88
14	82	0.112	1	0.58	164	0.25	1.70
**15**	**82**	**0.112**	**1.5**	**0.53**	**150**	**0.232**	**1.69**
16	82	0.246	0.5	0.76	185	0.28	1.95
17	82	0.246	1	0.72	174	0.272	1.87
18	82	0.246	1.5	0.68	162	0.256	1.83
19	116	0.06	0.5	0.59	198	**0.308**	2.50
20	116	0.06	1	0.53	172	0.298	2.45
21	116	0.06	1.5	0.45	165	0.272	2.42
22	116	0.112	0.5	0.61	210	**0.318**	1.79
23	116	0.112	1	0.54	195	**0.306**	1.77
24	116	0.112	1.5	0.44	183	**0.3**	1.75
**25**	**116**	**0.246**	**0.5**	**0.67**	**215**	**0.344**	**1.75**
26	116	0.246	1	0.65	207	**0.326**	1.71
27	116	0.246	1.5	0.62	201	**0.308**	1.51

The properties of graphene nanoparticles have been mentioned in Table 2. The graphene nano-particles have been blended into soybean oil in different concentrations using standard procedure. For the measurement of tool wear, machining time of 90 s has been fixed for all experiments and inserts have been examined under tool maker microscope for evaluation the of flank wear referring ISO3685. Nine cutting inserts of TNMG160408 type have been utilized for machining work piece under different conditions having 3 experiments on each inserts. The levels of machining parameters have been selected according to pilot survey, machine specification and expert opinion. Suitable numbers of repeatability has been maintained to ensure the reliability of experiment results. The L_27_ O.A has been used as DOE and ANOVA analysis has performed to optimize the experimental results. The setup utilized for machining, temperature measurement and surface roughness evaluation has been shown in Fig. 1. Also, the experimental planning for each trial has been illustrated in Fig. 2 visualizing machining time, work piece diameter and length of work piece. Suitable marking has been done on the work piece to distinguish the different machining conditions as visible in Fig. 2.

RETRACTED

**Fig. 1:** Photographic view of experimental setup.

**Fig. 2:** Plan of experiment on work piece.

Moreover, SEM of insert edges has been performed to identify the mechanism and intensity of tool wear at different section of insert. The coefficient of friction and shear angle have been computed on the basis of metal cutting theories like Ernest and Merchant formula. These factors have been introduced because the coefficient of friction (μ) explores the lubrication action, while the shear angle (φ) represents the behavior of material during machining. Lower coefficient of friction and higher shear angle are desirable for better machining performance. The tool wear has been measured with tool maker microscope, while the temperature is evaluated using digital infrared thermometer. Further, the surface roughness of worked component has been evaluated with digital roughness tester. The chip reduction coefficient ‘ζ’ (CRC) = tc/t has been calculated by measuring the chip thickness (tc) by digital vernier and uncut chip thickness t = f *Sin*Kr. Where f indicates feed rate and Kr is side cutting edge angle (93°). The shear angle has been evaluated by formula, φ $=\tan^{-1}\frac{rcos\alpha }{1-rsin\alpha }$ , coefficient of friction coefficient, μ=tanβ and β=90+φ−2α. Symbol r is ratio of chip thickness which is reciprocal of CRC, α is rake angle of tool and β is friction angle.

RETRACTED

### 2.1 Preparation of nano fluids

Blackish colour Graphene nano particles (GnP) of thickness 5–10 nm manufactured by Platonic Nanotech Pvt. limited India, has been utilized for research work. There are 4–8 numbers of layers in graphene as visible SEM image along with this, XRD analysis indicates the intensity of 90 Au having 2θ near to 25° visible in Fig. 3. The density of graphene nanoparticle is 150 kg/m^3^ and thermal conductivity of 2000 W/m-K. It has electrical conductivity of Siemen 10^7^/m and elastic modulus greater than 1000 GPa. The nano particles have been blended to 500 ml sample of soybean oil in different wt/vol. ratio like 0.5, 1 and 1.5% and mixed for 30 min in mechanical mixture. Further, Ultra sonication has been performed for 60 min then after magnetic stirring for 30 min. The homogenous mixture has been applied for heat dissipation and oiling during turning operation.

**Fig. 3:** SEM and XRD analysis of Graphene.

The properties of soybean oil and other mixtures have been measured using standard procedure and listed in Table 2. The viscosities and thermal conductivity of samples have been measured with digital viscometer set at 40 °C and transient hot wire apparatus. The observed values indicate that the flash point, specific gravity, kinematic viscosity and thermal conductivity increases with addition of graphene nanoparticles. The investigation into hard turning of Vanadis 10 examined that machining environment is most influential parameter to impact he surface roughness [54]. Also the optimization of EDM during processing of C22 superalloy revealed that peak current was major contributor for variation in surface roughness and MRR [55].

The addition of GnP has enhanced the thermal condctivity of sample by 4.09%, 7.01 and 12.28% as compared to pure soybean oil. In addition to this, the flash point has been increases by 3.33, 5% and 7.5% respectively. The same observation have been reported by Refs. [56,57]. Although, the viscosity has also been raised, but would be compenstaed by higher temperature during metal cutting at advanced level of process parameters. The photographic view of mixture preparation have been shown in Fig. 4, Fig. 5 (a-c) visualizing the nanoparticle container, weighing balance, ultrasonicator set up and magnetic stirring. The upmost care has been taken during preparation and application of samples to avoid any health issues.

RETRACTED

**Fig. 4:** Photographic view of grephene nano-particles, weighing balance and atomic Structure.

**Fig. 5:** Preparation of sample on Ultrasonicator and hot stirring.

Fig. 4d shows the photographic view and the atomic structure of graphene of nanoparticles in packaged form (Fig. 4a) and weighing balance (Fig. 4c) required to measure the mass of nanoparticle to be mixed with volume of soybean oil. Also, the setup used for Ultrasonication of sample along with hot stirring has been demonstrated in Fig. 5 (a-c) containing the sample of 500 ml per beaker. The open container consisting of blackish colour graphene nano-particles has been visualized in Fig. 4b.

The Wt/vol % of mixture has been calculated by formula mentioned in equation (1)**,** and the weight of nanoparticles has been increased in three steps 2.5 gm, 5 gm and 7.5 gm to obtain 0.5%, 1% and 1.5% of concentration of GnP in soybean oil.

(1) $$\frac{Wt.\;\left(gm\right)of\;nanoparticle\;\left(GnP\right)}{Vol.\;\left(ml\right)of\;soybean\;oil}*100=\frac{2.5\;gm}{500\;ml}*\;100=0.5\%$$

The apparatus used for recording of cutting temperature using infrared thermometer (Fig. 6a) and measurement of surface roughness have been displayed in Fig. 6 (b). Fig. 7a indicates the TNMG type insert followed by tool maker microscope Fig. 7b (Radical, RTM900DM) and photographic view of edge during measurement of flank wear Fig. 7c (see Fig. 8).

**Fig. 6:** (a) Display of infrared thermometer and (b) digital roughness tester.

**Fig. 7:** Tool wear of TNMG insert on tool maker microscope.

**Fig. 8:** Residual plot for S.R.

After experimental observation, the optimization of input variables has been carried out using ANOVA in MINITAB-11 and modelling equation has been formed for all responses.

## 3 Results and discussion

The outcomes of all 27 trials for surface roughness, cutting temperature, tool wear and chip reduction coefficient has been explored in Table 3. Further, the ANOVA analysis of input parameter and their percentage contribution on output responses have been extracted out. Also**,** the main effect and interaction charts have been drawn to explore the influence of each input variable on the outcomes. Moreover, two other responses like friction coefficient (μ) and shear angle (φ) have been calculated on the basis of CRC data utilizing fundamentals of metal cutting. Finally, the SEM analysis of worn inserts has been performed to find the mechanism and extent of wear.

### 3.1 ANOVA investigation for S.R

The analysis of variance (ANOVA) for S.R has been shown in Table 4 signifies that the model and input variables are valuable due to *P*-value shorter than 0.05. The S.R is greatly impressed by speed (41.66%) trailed by feed rate (28.16%) and then after concentration (13.68%). As the speed increases, the cutting forces reduces due to thermal softening of material which minimize the severity of BUE and thus makes the cutting process easier and henceforth produces good surface quality. Also, the concentration of nanoparticle into base oil play significant role to reduce the cutting forces in primary deformation zone. It is due to easy penetration (rolling and ploughing effect) of nanofluids to cutting zone and formation of lubrication layer makes the cutting easier, reduction in coefficient of friction and therefore, enhancement of surface roughness. However, increment in feed rate decline the surface quality due to higher chip load, BUE formation and causes the feed marks on the newly generated surface and consequently reduction in surface quality. Therefore, it is necessary to provide the cooling and lubrication at cutting zone to avoid the demerits of high friction, cutting forces and to maintain the sharpness of cutting edge. The author [21] has obtained the similar outcomes.

RETRACTED

**Table 4:** ANOVA summary for SR.

Analysis of Variance (ANOVA) for Surface roughness							
Source	DF	Seq SS	Contribution	Adj SS	Adj MS	F-value	*P*-value
Cutting speed A (m/min)	2	0.08436	41.66%	0.08436	0.042181	25.24	0.000
Feed rate B (mm/rev)	2	0.05703	28.16%	0.05703	0.028515	17.06	0.000
NC (%) C	2	0.02770	13.68%	0.02770	0.013848	8.28	0.002
Error	20	0.03343	16.51%	0.03343	0.001671		
Total	26	0.20252	100.00%				
Model Summary		**S**	**R**^**2**^	**R**^**2**^**(adj.)**	**PRESS**	**R**^**2**^**(Pred.)**	
		0.0408838	83.49%	78.54%	0.0609255	69.92%	

In addition to this, the R-square and adjusted R-square are close to each other having values greater or near to 80%, which is desirable for better results as per statistical analysis. The empirical equation for S.R obtained from analysis has been described in equation (2).

(2) S.R(Ra)μm=0.63259+0.0707*A(m/min)_51−0.0048*A(m/min)_82−0.0659*A(m/min)_116−0.0415*B(mm/rev)_0.060−0.02268*B(mm/rev)_0.112+0.0641*B(mm/rev)_0.246+0.0419*(Conc%)_0.5−0.0059*C(Conc%)_1.0−0.0359*C(Conc%)_1.5

### 3.2 Analysis of variance for temperature

The ANOVA Table 5 for temperature indicates that cutting speed is dominant to influence the temperature majorly (69.31%), afterward concentration (14.53%) and feed rate (13.25%). It means the higher cutting speed generates excessive friction that will negatively affect the cutting edge of tool and thus degrade the quality of generated surface.

**Table 5:** ANOVA summary for temperature.

Analysis of Variance (ANOVA) for temperature							
Source	DF	Seq SS	Contribution	Adj SS	Adj MS	F-value	*P*-value
Cutting speed A (m/min)	2	10724.5	69.31%	10724.5	5362.26	237.58	0.000
Feed rate B (mm/rev)	2	2049.9	13.25%	2049.9	1024.93	45.41	0.000
NC (%) C	2	2247.6	14.53%	2247.6	1123.81	49.79	0.000
Error	20	451.4	2.92%	451.4	22.57		
Total	26	15473.4	100.00%				
Model Summary		**S**	**R**^**2**^	**R**^**2**^**(adj.) (adj.)**	**PRESS**	**R**^**2**^**(Pred.)**	
		4.75083	97.08%	96.21%	822.69	94.68%	

Therefore, it is necessary to minimize the excessive rubbing and heat formation during turning of material (Hastelloy C-276) having low thermal conductivity by the application of nanoparticles that absorb the intense heat due to impingement in the cutting zone and hence provide the cooling effect. Thus, maintain the sharpness of cutting edge and cut the material smoothly, sustain good surface finish, and longer tool life. Moreover, increase in level of feed rate hike the temperature because of higher chip load on cutting insert. The main reason behind the elevated temperature at higher levels of v is due to friction and rubbing at tool chip interface. Moreover, increment in feed rate causes higher chip load and friction leading to higher temperature. Regression equation for temperature is given by

(3) Temp(°C)=167.852−22.19*A_51−3.96*A_82+26.15*A_116+10.85*B_0.060+0.37*B_0.112+10.48*B_0.246+10.93*C_0.5+0.48*C_1.0−11.41*C_1.5

The terms R^2^ and R^2^ (adj.) are adjacent (97% and 96%) to each other signifies the accuracy of developed model with experimental results. The regression equation for temperature is listed in equation (3). The heat absorption capacity of GnP along with lubrication ability of soybean oil minimize the temperature and thus have more influence on heat generation than feed.

RETRACTED

### 3.3 ANOVA for tool wear

The ANOVA Table 6 for tool damage designate that cutting speed is supreme factor (67.2%) to influence tool wear due to production of large temperature and intense friction causing damage on tool surface. In addition to this, higher speed generates excessive rubbing at tool-chip and tool work interface that leads to damage on flank and crater portion of cutting tool. The similar outcomes have been listed by Ref. [17].

**Table 6:** ANOVA Summary for tool wear.

Analysis of Variance (ANOVA) for Tool wear							
Source	DF	Seq SS	Contribution	Adj SS	Adj MS	F-value	*P*-value
Cutting speed A (m/min)	2	1.23796	67.20%	1.23796	0.618978	173.44	0.000
Feed rate B (mm/rev)	2	0.44027	23.90%	0.44027	0.220133	61.68	0.000
NC (%) C	2	0.09260	5.03%	0.09260	0.046300	12.97	0.000
Error	20	0.07138	3.87%	0.07138	0.003569		
Total	26	1.84220	100.00%				
Model Summary		**S**	**R**^**2**^	**R**^**2**^**(adj.) (adj.)**	**PRESS**	**R**^**2**^**(Pred.)**	
		0.05974	96.13%	94.96%	0.130086	92.94%	

Further the sticking and sliding zone in Primary deformation section (tool-chip interface) impact the tool wear due to intensive friction and continuous contact causing adhesion, abrasion and diffusion type of wear. Secondly, feed rate have altered the flank as well crater section of insert significantly with contribution (23.90%) because of expansion in chip load, expanded tool chip contact length which is producing higher rubbing at these section. Further, to check the predicted and actual outcomes the empirical relation for tool wear is given by equation (4).

(4) ToolWear(mm)=1.2533−0.2178*A_51−0.0733*B_82+0.2911*B_116−0.1711*B_0.060+0.0356*B_0.112+0.1356*B_0.246+0.0700*C_0.5+0.0033*C_1.0−0.0733*C_1.5

The contribution of nanoparticles concentration on tool wear is significant (5.03%) due to absorption of heat and subsequent lubrication effect of vegetable oil accompanying air jet cooling. Further, the statistical terms like R-square and adjusted R square adjacently indicates that the predicted and experimental results fit well.

### 3.4 Statistical plots for output responses

The statistical plots indicate the relation between predicted results and experimental observations. The accuracy of developed model can be verified from Residual plots having charts like Normal Probability, residual vs. fitted values, frequency and observation order of residual. In these types of plots, the confidence level of 95% can be verified from normal probability graph, whereas the predicted vs. experimental results can be confirmed from residual vs. fitted value chart. Moreover, the frequency of residual along with observation order can be checked that indicates the deviation from mean line. **The Plot 8** indicates that majority of the values are lying on the line and the residual are falling within the uniform range of 0.10.

Similarly, the Normal probability plot for cutting temperature shown in Fig. 9 has maximum spots clinging to straight line suggest the accuracy of predicted and observed values of cutting temperature. Moreover, the scatter of points visible in Fig. 10, Fig. 11 also illustrates the significance of regression equation generated for tool wear and CRC. From all these plots, it has been confirmed that experimental and predicted results of all the responses lies within 95% confidence limit.

**Fig. 9:** Statistical plots for temperature.

**Fig. 10:** Statistical Plots for tool wear.

**Fig. 11:** Statistical plots for CRC

The residual plots for coefficient of friction and shear angle have been depicted in Fig. 12, Fig. 13 illustrates that the predicted as well as observed values are very close to each other. Further, the normal probability plots for both indicates that the scatter of data adhere to line, which suggest 95% confidence limit and accuracy of developed model. In addition to this, Fig. 12 indicates that only 33% values of friction coefficient are more than 0.5 and contrary to this, 67% values of shear angle (Fig. 13) are less than 27°. It revealed that lower coefficient of friction and higher shear angle among experimental observation have been reported and hence obtained outcomes are desirable as per literature studies [21,22].

RETRACTED

**Fig. 12:** Statistical Plots for coefficient of friction (μ).

**Fig. 13:** Residual plot for Shear angle (φ).

### 3.5 Main effect plot for output responses

The effect of all input variables on output responses have been illustrated in Fig. 14, Fig. 15, Fig. 16. Fig. 14 (a) indicates that the surface quality of specimen diminish with rise in feed rate owing to larger chip load on cutting edge of tool and higher tool chip contact length on the nose part. While, the nanoparticles concentration has minimized the roughness due to heat absorption, penetration of GnP to cutting zone together with favorable lubrication action of oil that provide the cushion effect and maintain the sharpness of cutting edge. Fig. 14 (b) represents that the cutting temperature rises directly with speed due to involvement of friction at various sections of tool-work piece interaction. As visible in Fig. 14 (a), the surface roughness reduces on hike of cutting speed due to thermal softening of specimen and reduction in cutting forces at different zones of metal cutting. Consequently, cuts the material softly and produces the better surface quality.

**Fig. 14:** Influential impression plot for SR and Temperature.

**Fig. 15:** Main effect plot for tool wear and CRC.

**Fig. 16:** Main effect plot for friction coefficient (μ) and Shear angle (φ).

The metal cutting is very complex because of minor contact of the tool-work, tool chip and very less time of interaction at various sections of deformation. Thus, in this short period of time numbers of parameters are active and should be carefully considered for better experiments observation in line with theoretical results. The variation of feed rate also escalates the temperature linearly as mentioned earlier due to jump in chip load and more area of cutting ahead of cutting tool. However, increment in nanoparticle concentration reduces the temperature because of heat absorption effect along with lubrication film of bio-oil and cooling ability of air assisted jet jointly. This is only the factor which has diminished the surface roughness, heat generation, tool damage and CRC compared to other. Similarly, tool wear become rapid on increasing the speed and feed rate due to higher friction and more chip load. Unlike this, it reduces on increasing the concentration on nanoparticles mixed with vegetable based oil and is visible in Fig. 15 (a). On the other hand, CRC have different behaviour as compared to other variables during variation of input variables. CRC increases first and then reduces while cutting speed is changed as shown in Fig. 15 (b). Along with this, it also reduces with increase in feed rate as well as nanoparticle concentration. The reason behind the same is due to variation in chip thickness, reduction in cutting forces at interface because of rolling, mending and tribo-film formation along with lubrication action of vegetable oil. All these effects can reduce the friction coefficient as well causing reduction in CRC.

RETRACTED

Fig. 16 (a) specifies that the coefficient of friction (μ) expand initially on surging the cutting speed and then decline. It is due to change in temperature and nanoparticle concentration that impact the friction coefficient. However, reverse results has been obtained for shear angle (φ) compared to friction coefficient are depicted in Fig. 16 (b). During starting phase of cutting, (φ) reduces and then increases with increment in v due to change in cutting forces, heat generation and friction coefficient. However, it rises with increase in f due to change in chip thickness and frequency of chip formation. Moreover, there is downward trend of friction coefficient with rise in nanoparticle concentration due to heat absorption, rolling and tribofilm-cushion effect of vegetable oil GnP-air jet amalgamation during cutting operation. The 2D foil micrograph of graphene nanoparticles have weak Vandar wall forces between the layer and easily shearing led to provide tribo-layer on the surface of tool and thus reduces insert erosion as well as friction coefficient. Also, the application of nano-MQL to tool-chip interface reduces the tool-chip contact length and thus reducing the coefficient of friction because of rolling, mending and ploughing effects of GnP. In addition to this, the heat absorption capacity increases as the concentration of nanoparticle due to rise in conductivity of mixture as listed in Table 4. Also, the viscosity of nano-fluids decreases with rise in temperature and hence lower viscosity is required for easily flowing of mixture during application MQL for pumping power requirement. The concentration of nano particle can be increases up to certain limit to avoid problems of aerosol flow, ploughing effect (causing wear of tool and higher roughness) and may choke the MQL nozzle. Also from literature survey, it has been learned that the concentration more that 2.5 w/v concentrations can give rise to tool wear. Therefore, the pilot tests were conducted to confirm these limits and hence only these three types of concentration have been chosen. Also, addition of nanoparticle can impact the free energy of liquid-solid and air interface and changes the contact angle which further inflates the wetting of tool surface and hence increases the cooling ability of amalgamation. The lower contact angle is always desirable for excellent wetting ability and consequently more cooling action at tool chip interface.

RETRACTED

### 3.6 Contour plots for output responses

The contour plots have been shown in Fig. 17, Fig. 18, Fig. 19, Fig. 20, so as to identify the best range of input factors having better performance of output variables. Fig. 17 (a, b) signifies that lower surface roughness noticed at v of 95–115 m/min along with f of 0.06–0.14 mm/rev and nanoparticle concentration 1.20–1.50%. Since, higher speed, lower feed and more concentration of nanoparticles resulted into better surface quality as mentioned earlier.

**Fig. 17:** effect of cutting speed, feed rate and NC on SR.

**Fig. 18:** Effect of cutting speed, feed rate and NC on cutting temperature.

**Fig. 19:** Impact of speed, feed and NC on tool wear.

**Fig. 20:** Impact of cutting speed, feed rate and NC on coefficient of friction (μ).

As depicted in Fig. 18 (a) the lower cutting temperature (<160 °C) have been achieved at 90 m/min together with all levels of feed rate. Contrary to this, higher cutting temperature has been recorded after 95–115 m/min at ‘f’ 0.07 mm/rev**.**

The less temperature (Fig. 18 b) has been observed at concentration of 1.25–1.5% having cutting speed of about 60 m/min. Investigation disclosed that the speed range of 60–90 m/min, temperature of 160–180 °C has been maintained by lower level of nanoparticle concentration.

. All these observation revealed that rise in cutting speed accelerate the temperature due to increment in friction at cutting zone and higher concentration reduces the heat generation because of combined cooling and lubrication effect of GnP nano MQL. These outcomes support the literature data [[22], [23], [24]]. As shown in Fig. 19 (a), lower tool wear has been noticed at 60–90 m/min along with 0.06–0.09 m/min feed. However, tool life ends quickly beyond 110 m/min along with feed rate 0.10 mm/rev and 1.25% nanoparticle concentration. This is caused by the combined effect of both ‘v-f’ as visible in Fig. 19 (a, b). Further from Fig. 19 (b) it is clear that maximum area has been covered by concentration in speed range of 84–95 m/min give the best tool life and lower wear.

RETRACTED

Fig. 20 (a, b) signifies that lower coefficient of friction have been reported at 0.12–0.22 mm/rev feed along with NC of more than 0.75%. On the other side, higher shear angle has been reported at speed range of 80–110 m/min accompanying ‘f’ 0.14–0.22 mm/rev (Fig. 21 a). Likewise, larger shear angle (φ) has been noticed from Fig. 21 (b) at concentration of 0.75–1.5% having speed rate of 92–110 m/min.

**Fig. 21:** Impact of cutting speed, feed rate and NC on shear angle (φ).

This has been happened due reduction in cutting forces with rise in speed as discussed earlier because of tribo film formation and exploration of nanoparticle layer into deformation zone, lubrication effects of vegetable oil and self-lubrication ability of graphene molecules. Also, the reduction in CRC is the indicator of lower cutting force in deformation due to thermal softening and lower severity of BUE. Further, the reduction in viscosity also played a major role in minimization of coefficient of friction and thus produces favorable machining conditions. The larger shear angle indicates the easier machining condition and lower power requirement.

### 3.7 Interaction plots for output responses

The interaction plot examines the influence of input variables on out responses. In present investigation Fig. 22, Fig. 23, Fig. 24 shows impact of various input parameters on output responses. The main effect plot shown earlier indicates only the overall impact and the behaviour of individual factor. However, this type of plot signifies the effective range of input variables.**.**

**Fig. 22:** Interaction plot for SR.

**Fig. 23:** Interaction plot for Temperature.

**Fig. 24:** Interaction plot for tool wear.

Fig. 22 illustrates that minimum SR have been reported at 116 m/min velocity, 0.112–0.116 feed and 1.5% of GnP concentration. Similarly, less cutting temperature has been found at ‘v’ 51 m/min together with 0.06 mm/rev and 1.5% of NC as visible in Fig. 23.

Cryogenic treatment of AISI O_2_ cold worked steel utilizing coated and uncoated tool having Taguchi L_16_ was used to optimize the levels of speed, feed and tool types for enhancing the surface roughness [58]. Hence, careful selection of parameters is necessary for economic of machining. Also, Taguchi optimization of surface roughness and tool wear while machining DIN 1.2344 (Turning), Hardox 400 steel (Milling) revealed that feed rate was dominant input variable. The significant levels of cutting speed and feed rate were found as 120 m/min and 0.15 mm/rev [59,60]. Similar trends have been found in present investigation as well shown in Fig. 22.

RETRACTED

The lower tool wear has been noticed during 1.5% of NC at ‘v’ 51 m/min and feed of 0.060 mm/rev in Fig. 24. It is because of better cooling action, enhanced heat absorption capacity of nanoparticle mixed with vegetable oil lubricant [[61], [62], [63]]. The application of GnP and vegetable oil reduces the tool chip contact length resulting into minimization of heat generation due to reduction in friction at tool chip interface because of GnP rolling action and lubrication film of vegetable oil [[64], [65], [66]]. These entire cooling and lubrication phenomenon boost the surface finish, tool life, CRC and friction coefficient [[67], [68], [69]].

Further, the minor value of CRC is highly recommended to have lower cutting forces and power requirement. Hence, minimum CRC has been reported at 0.246 mm/rev and 116 m/rev in Fig. 25. There is minor variation in CRC during 0.06 and 0.112 mm/rev and the percentage contribution of ‘f’ is very high as compared to other parameters due to the complexity of cutting conditions. It is owing to change in uncut chip thickness which influence the CRC as f varies. Moreover, the lower coefficient of friction has been found during 116 m/min, 0.246 mm/rev and 1.5% NC as depicted in Fig. 26. On the other side**,** higher value of shear angle is recommended for favorable machining conditions and for present research the shear angle has been found large at 116 m/min speed with ‘f’ value 0.246 mm/rev and 1.5% concentration of GnP (Fig. 27). From all these scenarios of experimental results, it can be revealed that higher concentrations of nanoparticle have fulfilled the objective function for minimization of temperature, roughness, tool wear, CRC and coefficient of friction [[70], [71], [72]]. Moreover, the objective to maximize the shear angle has also been achieved at 1.5% NC.

**Fig. 25:** Interaction plot for CRC.

**Fig. 26:** Interaction plot for Coefficient of friction (μ).

**Fig. 27:** Interaction plot for shear angle (φ).

### 3.8 SEM analysis of tool wear

In present investigation, the SEM apparatus manufactured by JEOL has been utilized for evaluation of tool wear and its mechanism. Fig. 28 (a) illustrates the SEM image of fresh carbide insert edge in which there are no sign of deformation on the rake as well as flank sections of an insert. However, in Fig. 28 (b), nose wear, abrasion, adhesion and loss of coating and flank wear of 0.221 mm have been reported during 82 m/min, 0.112 mm/rev and 1.5% NC concentration of graphene nanoparticle. This phenomenon has occurred due to chip rubbing at rake face and friction between flank and freshly generated work surface [[73], [74], [75]].

**Fig. 28:** **(a)** SEM image of unused insert edge; **(b)** 82 m/min, 0.112 mm/rev and 1.5% NC.

RETRACTED

In addition to this, the material adhesion is due to chemical affinity of tool material and lower thermal conductivity of workpiece which should be minimized by application of suitable cooling and lubrication media [[76], [77], [78]]. The higher friction at tool face causes the softening of tool material leading to reduction in its hardness causing the physical removal of tool material from parent material, cracks, quick plastic deformation, more cutting forces and as a result crater wear and premature failure (Goindi and Sarkar 2017). Moreover, the nanoparticles concentration has direct influence on the tool wear that absorb the heat and reduced the adhesion on the rake portion of insert and thus reduces tool damage [[79], [80], [81]]. However, friction due to sliding and rotary motion of chip has created the abrasion marks on the top surface of cutting tool where the lubricant media is not accessible due to high sliding velocity and lower cutting area. Hence, dual lubrication nozzle should be the good option for to reduce the same [[82], [83], [84]].

The severity of damage on nose, flank and crater sections of the tool has been illustrated in Fig. 29 (a). The magnitude of flank wear 0.172 mm has been reported during these machining conditions and same has been visible in Fig. 29 (a). The main reason behind little tool erosion than previous case is due to smaller v, f and higher accumulation of nanoparticles (1%) [[85], [86], [87]]. However, few spots of adhesion, breakage of nose part along with abrasion marks have been reported [[88], [89], [90]]. Finally, the larger flank, crater wear accompanying nose damage and complete failure of tool have been reported during 116 m/min, 0.246 mm/rev having 0.5% NC illustrated in Fig. 29 (b).

**Fig. 29:** **(a)** SEM micrograph at 51 m/min, 0.06 mm/rev and 1% NC; **(b)** 116 m/min, 0.246 mm/rev and 0.5% NC.

During these machining condition impaired surface roughness (0.67 μm), intense cutting temperature (215 °C), rapid flank wear (344 μm) and 1.75 CRC have been observed. It has happened due to higher intensity of v, f and lower nanoparticle concentration. The experimental results of tool wear have been found satisfactory with SEM analysis at various levels of input parameters.

From Fig. 30, it is clear that tool life ends at higher level of input parameters (116 m/min) during all feed condition having concentration of 0.5 and 1%. However, there is only one situation during 1.5% NC at which tool failure occurred. The experimental results revealed that tool failure occurred 6 times out of 27 trials and depicted in blue, red and green colour at 116 m/min as visible in Fig. 30. In addition to this**,** it has been observed that tight coiled spring form of chip have been produced during all machining conditions [91,92].

RETRACTED

**Fig. 30:** Analysis of tool wear at 0.5 mm doc and 90 s of machining time.

### 3.9 Mechanism of metal cutting, heat generation, cooling and lubrication effect

The metal cutting is very complex in nature due to different deformation zones, minor contact of tool-work and tool-chip along with high frequency of chip formation and numerous forces at different sections [93,94]. The thermal state of turning operation and the classical model of metal cutting has been shown in Fig. 31, Fig. 32 demonstrating the workpiece, cutting tool, different deformation zones, chip formation, rake and flank face. In addition to this, MQL nozzle comprising of GnP blended with vegetable oil targeted at the rake face of cutting tool along with graphics of rake and shear angle has been demonstrated in Fig. 32. In primary deformation zone (PDZ), the direct contact of cutting tool and work material leads to compressive, shearing and ploughing type of elasto-plastic deformation producing heat due to breaking of material bond [95]. Various types of chips are produced in this section depending upon the ranges of process parameters, material and lubrication conditions. On the other hand, in secondary deformation zone (SDZ), the plastic deformation, sticking-sliding friction between the generated chip and rake face of tool produces high temperature at interface of primary and secondary zone [96,97].

**Fig. 31:** Thermal state of metal cutting zones in turning.

**Fig. 32:** Mechanism of metal cutting using Gnp nano-MQL.

Consequently, erode the tool material and impact the cutting forces as well as surface quality. Moreover, in tertiary deformation zone (TDZ), the elastic deformation and friction between newly developed surface affect the flank wear [97,98]. Hence, there is a requirement to reduce the friction at tool chip and tool work interface to minimize the surface roughness, cutting forces and tool wear. The same can be possible with the aid of suitable cooling and lubrication media focused at different zones of deformation [99,100].

The mechanism of nano-MQL cooling and lubrication action has been expanded in Fig. 33, Fig. 34. It should be noted that the maximum amount of heat generated in primary deformation zone (60–65%) is carried away by the chip; 30–35% of supplied energy in converted into heat in SDZ and about 5–10% of energy is converted into heat in TDZ [95]. Hence, it is of upmost significance to reduce the severity of friction at different section of deformation during turning of Hastelloy C-276 for which low thermal conductivity creates the problem of quick tool wear.

RETRACTED

**Fig. 33:** Mechanism of nano-MQL cooling.

**Fig. 34:** Mechanism of lubrication.

The GnP-MQL focused on the rake face of tool provide the cooling and lubrication action at the different deformation zones due to higher thermal conductivity of graphene nanoparticles that absorb the heat and form the tribo-film due to hexagonal atomic structure enabling the rolling effect in cutting zone [[101], [102], [103]].

Also, the bio-based oil provides the lubrication action due to atomized droplets striking into asperities of deformation at primary and secondary zone as illustrated in Fig. 35, Fig. 36.

**Fig. 35:** Mechanism of GnP nano-MQL Lubrication in different zones.

**Fig. 36:** Comparison of contact angle [57].

The dual cooling and lubrication action of airjet, GnP and vegetable oil is able to reduce the friction, cutting forces and thus enhances the surface roughness, tool wear and shear angle. Moreover, the utility of GnP has high thermal conductivity that absorb the heat effectively and produces more wetting of contact surface due to reduction in contact angle.

However, in sticking zone the lubrication effect is not much superior due to permanent contact of tool-chip for small interval of time and thus increases the wear rate on the rake face of tool [104,105]. On the other hand, the impingement of GnP-nano MQL in TDZ produces the handsome cooling and lubrication action and hence lower flank wear as compared to rake face [106,107]. The same effect has also been observed in SEM image shown in Fig. 29, Fig. 30 indicating the more wear on the rake face as compared to flank part. Finally, it has been concluded that higher concentration (1.5%) of GnP-nano MQL has minimized the friction, cutting forces, surface roughness and tool wear effectively leading to enhancement of machining performance significantly compared to lower concentration.

## 4 Conclusions

### 4.1 From all experimental investigation, it has been revealed that

i. The addition of GnP in different concentration (0.5, 1 and 1.5%) has enhanced the thermal conductivity of sample by 4.09%, 7.01 and 12.28% as compared to pure soybean oil. In addition to this, the flash point has been increases by 3.33, 5% and 7.5% respectively.
ii. The surface quality is superimposed by speed rate (41.66%) trailed by feed rate (28.16%) and then after concentration (13.68%). Temperature is dominated by cutting speed (69.31%), afterward concentration (14.53%) and feed rate (13.25%). Likewise, tool wear has been majorly altered by speed (67.2%) afterward feed rate (23.90%) and thirdly concentration of GnP (5.03%). Whereas, CRC has been accomplished 79% by feed rate and 4% during cutting speed and concentration both.
iii. Good surface finish reported at higher levels of speed, lower ranges of feed and maximum concentration of nanoparticles. Whereas, least cutting temperature has been reported at initial levels of speed accompanying the all levels of feed rate.
iv. Less tool wear has been noticed at speed level of 60–90 m/min accompanying feed rate of 0.06–0.09 m/min. However, tool life ends quickly beyond 110 m/min along with feed rate of 0.10 mm/rev.
v. The output parameters like temperature, surface roughness, CRC, tool wear, friction coefficient (μ) and shear angle have been influenced by the concentration (0.75–1.5%.) of GnP greatly.
vi. Utilization of 1.5% GnP concentration has reduced the roughness (11.47%–27.88%), temperature (6.5%–16.8%), tool wear (6.12%-22.5%), CRC (3.75–17.5%), coefficient of friction (7.05–46.36%) and shear angle (4–15%) compared to other.
vii. SEM analysis indicated nose wear, abrasion, adhesion and loss of coating. The flank wear of 0.221 mm has been reported at 82 m/min, 0.112 mm/rev and 1.5% NC. Whereas, complete failure of tool has been reported during 116 m/min, 0.246 mm/rev having 0.5% NC.

RETRACTED

## Author contribution statement

Gurpreet Singh: Conceived and designed the experiments; Performed the experiments; Analyzed and interpreted the data; Wrote the paper.

Shubham Sharma: Conceived and designed the experiments; Performed the experiments; Analyzed and interpreted the data; Contributed reagents, materials, analysis tools or data; Wrote the paper.

A.H. Seikh: Yanbin Zhang: Rajesh Singh: Sayed M. Eldin: Analyzed and interpreted the data; Contributed reagents, materials, analysis tools or data.

Changhe Li: Abhinav Kumar: Analyzed and interpreted the data; Contributed reagents, materials, analysis tools or data; Wrote the paper.

S. Rajkumar: Performed the experiments; Analyzed and interpreted the data; Contributed reagents, materials, analysis tools or data.

## Data availability statement

Data included in article/supp. material/referenced in article.

## Declaration of competing interest

The authors declare that they have no known competing financial interests or personal relationships that could have appeared to influence the work reported in this paper. The authors declare that they have no conflict of interest with respect to the research, authorship, and/or publication of this article. The authors don’t receive any research fund or grant from any organization. This article does not contain any studies with human participants or animals performed by the author.
